# Associations of Urinary Phytoestrogen Concentrations with Nonalcoholic Fatty Liver Disease among Adults

**DOI:** 10.1155/2022/4912961

**Published:** 2022-03-31

**Authors:** Guang Xiong, Changbo Huang, Yuping Zou, Ziyin Tao, Jun Zou, Jiean Huang

**Affiliations:** Department of Gastroenterology, The Second Affiliated Hospital of Guangxi Medical University, Nanning 530007, China

## Abstract

Phytoestrogens can alleviate some pathological processes related to nonalcoholic fatty liver disease (NAFLD). However, there are limited and contradictory studies on the relationships between phytoestrogens (especially single phytoestrogen) and NAFLD. The purpose of this study was to explore the relationships between urinary phytoestrogen concentrations and NAFLD in American adults. This cross-sectional study used the data of the National Health and Nutrition Examination Survey from 1999 to 2010, and 2294 adults were finally enrolled in this study. The concentrations of phytoestrogens were measured in urine samples, and urinary phytoestrogens were divided into tertiles according to the concentration distributions. The diagnosis of NAFLD was determined by the United States fatty liver index. The main analysis used a multivariate logistic regression model. The fully adjusted models included gender, age, race, education, marriage, poverty, body mass index, waist circumference, smoking, diabetes, hypertension, total cholesterol, high-density lipoprotein cholesterol, triglycerides, and other five phytoestrogens. In the fully adjusted model, the urinary enterolactone (ENL) concentration was negatively correlated with NAFLD (OR of Tertile 3 : 0.48, 95% CI 0.25–0.94). When stratified by age and gender, the urinary ENL concentration was negatively correlated with NAFLD in males aged 40–59 years (OR of Tertile 3 : 0.08, 95% CI 0.01–0.82), while the urinary equol concentration was positively correlated with NAFLD in such population (OR of Tertile 3 : 4.27, 95% CI 1.02–17.85). In addition, a negative correlation between enterodiol (END) concentration and NAFLD was observed in males aged 60 years or over (OR of Tertile 2 : 0.18, 95% CI 0.05–0.69). Collectively, in middle-aged males, urinary ENL may be associated with a lower risk of NAFLD, while urinary equol may be related to a higher risk. In addition, urinary END has a possible relationship with a reduced risk of NAFLD in elder males. Definitely, clinical randomized controlled trials are needed to further verify the conclusions.

## 1. Introduction

The incidence of nonalcoholic fatty liver disease (NAFLD) has been increasing year by year, and it has gradually become the leading cause of chronic liver disease worldwide [1, 2]. NAFLD can progress to nonalcoholic steatohepatitis, liver cirrhosis, and even hepatocellular carcinoma [3–6]. In addition, this disease is closely related to diabetes, cardiovascular disease, and chronic kidney disease and thus increases the risk of these diseases [7–12]. NAFLD is now considered to be a multisystem disease, which not only damages the liver itself but also affects multiple extrahepatic organs [8, 12]. Given its harmfulness, the need to prevent and treat NAFLD is apparent.

Phytoestrogens are a group of compounds produced by plants, which can mimic or interact with estrogens [13]. Because of their structural similarity to estrogens, they have estrogen/antiestrogen and antioxidant activities [14–16]. Phytoestrogens ingested by the human body mainly include two categories: isoflavones (mainly from soybean) and lignans (mainly from oilseeds, whole wheat, seeds, and nuts) [15, 16]. Isoflavones determined in the National Health and Nutrition Examination Survey (NHANES) are daidzein, O-desmethylangolensin (O-DMA), equol, and genistein. Daidzein can be metabolized into O-DMA and equol via the action of intestinal bacteria [17, 18]. The lignans measured in NHANES are enterodiol (END) and enterolactone (ENL) which are the metabolites of END [19, 20].

Studies have found that phytoestrogens have protective effects on many pathological processes related to NAFLD, such as regulating hepatic lipogenesis, improving insulin resistance, and promoting lipolysis [21, 22]. Although many animal experiments showed that isoflavones could reduce hepatic steatosis [23–26], there is a lack of relevant human research. Dietary isoflavone intake was negatively correlated with NAFLD in an observational study [27], and isoflavone supplementation improved insulin resistance in patients with NAFLD in a clinical trial [28]. The relationship between lignans and NAFLD has not been reported in human participants so far; only a few animal experiments have evaluated the association between lignans and hepatic steatosis, and there is no unified conclusion at present [29–34]. Furthermore, assessment of dietary phytoestrogens is difficult to cover all food sources and the metabolic transformation of phytoestrogens in the human intestine was not under consideration in the assessment, thus failing to accurately reflect real individual exposure. Hence, a measurement of urine concentrations of phytoestrogens will be required to reflect the real exposure. The purpose of this study is to explore the relationships between urinary phytoestrogen concentrations and NAFLD in American adults through NHANES, a large population cross-sectional survey, and further investigate the relationships in different genders and ages.

## 2. Materials and Methods

### 2.1. Study Samples

The subjects and data of this study were all enrolled and collected from NHANES, an ongoing cross-sectional, multistage, stratified probability sampling survey [35]. The survey is conducted by National Center for Health Statistics (NCHS), with NCHS Research Ethics Review Board approval and informed consent provided by all participants. We combined six-cycle data (NHANES 1999–2000, 2001–2002, 2003–2004, 2005–2006, 2007–2008, and 2009–2010) to create the samples for this study because urinary phytoestrogen concentrations were measured only in 1999–2010.

A total of 62160 subjects were included in the evaluation, and 32464 of them aged 20 years and over were selected. Then, 28906 participants who met the following criteria were further excluded [1]: (1) excessive alcohol drinking (>21 standard drinks per week for males and >14 standard drinks per week for females) (*n* = 845); (2) positive serology for hepatitis B or C virus (*n* = 619); (3) taking medications that can affect hepatic steatosis (*n* = 964); (4) taking gonadal hormone (*n* = 186); (5) self-reported cancer (*n* = 2628); (6) pregnant women (*n* = 1246); (7) missing information required for the definitions of NAFLD (*n* = 15285); and (8) missing data regarding phytoestrogens (*n* = 7133). After exclusion, 3558 participants were left, and we defined NAFLD by the United States fatty liver index (USFLI, see below for details). Ultimately, 1066 participants were considered to have NAFLD, and 1228 participants were divided into the non-NAFLD group (Figure 1).

### 2.2. Definition of Variables

We used USFLI which is a noninvasive method to define the presence of NAFLD [36]. The USFLI is calculated by weighting several indexes such as race, age, gamma glutamyltransferase, waist circumference, fasting insulin, and fasting blood glucose. The USFLI shows a good correlation with ultrasound-diagnosed NAFLD, which has been validated in a previous study [36]. As results of the study suggested, a USFLI score ≥30 was used to identify the presence of NAFLD, and a USFLI < 10 was considered to rule out NAFLD (Figure 2).

Participants who met one or more of the following criteria were defined as having diabetes [37]: (1) a diagnostic history of diabetes; (2) taking antidiabetic medications or insulin; (3) fasting blood glucose ≥126 mg/dl; and (4) hemoglobin A1c ≥ 6.5%.

Hypertension was defined as meeting one or more criteria [38], which include the following: (1) a diagnostic history of hypertension; (2) systolic blood pressure ≥140 mmHg and/or a diastolic blood pressure ≥90 mmHg; and (3) taking medicine to lower blood pressure.

### 2.3. Measurement of Urinary Phytoestrogens

The collection of urine samples and the determination of phytoestrogen concentration were carried out in mobile examination centers. The concentrations were determined by high-performance liquid chromatography-tandem mass spectrometry in the survey 1999–2004 and by high-performance liquid chromatography-atmospheric pressure photoionization-tandem mass spectrometry in the survey 2005–2010 [39]. After comparing the two methods, the NHANES research team demonstrated that the correlation coefficients of the results analyzed by the two methods was very high (*r* > 0.99), and the regression slopes approximately equaled to 1, and the intercept was close to 0 [39]. The experimental research manual provided a more detailed analysis process [40, 41]. According to many studies, urinary phytoestrogen concentrations can be used as a reliable biomarker of phytoestrogen intake [42–46]. Because the concentrations of markers in urine is easily affected by urine volume, the concentrations of urinary phytoestrogen were standardized with creatinine and expressed as ng/mg creatinine [47].

### 2.4. Covariates

The potential covariates included gender, age, race, education, marriage, poverty, body mass index (BMI), waist circumference, smoking, diabetes, hypertension, triglycerides, total cholesterol, and high-density lipoprotein cholesterol, which were selected to control confounding effects through the prior published studies [48–55].

### 2.5. Statistical Analysis

The complex stratified sampling design adopted by the NHANES could better reflect the overall situation of the population, so we used stratification, clustering, and an appropriate sample weight to carry out this study according to the NHANES analysis guidelines [56]. Data are expressed as the weighted mean ± standard error or weighted frequency (95% confidence intervals). The characteristics of the study population were compared between the NAFLD group and the non-NAFLD group. The differences of continuous variables were compared by one-way analysis of variance or the Kruskal–Wallis test, and the differences of classified variables by the chi-square test. Phytoestrogens were divided into tertiles according to the concentration distributions in the population. Multivariate logistic regression was used to analyze the relationship between urinary phytoestrogen concentrations and NAFLD. Model 1 adjusted the other five phytoestrogens. To further explore the relationship between them, model 2 increased demographic variables (gender, age, race, education, marriage, poverty) compared with model 1. Model 3 further adjusted all potential variables (BMI, waist circumference, smoking, diabetes, hypertension, triglycerides, total cholesterol, high-density lipoprotein cholesterol) on the basis of model 2. All tests in this study were two-sided tests, and *P* < 0.05 was considered significant. All data were processed using EmpowerStats (https://www.empowerstats.com, X&Y Solutions, Inc., Boston, Massachusetts) and statistical software package R (https://www.R-project.org; The R Foundation; version 3.6.3).

## 3. Results

### 3.1. General Patient Information

In total, 2294 participants were included in the analysis. The baseline characteristics of the NAFLD group and the non-NAFLD group are shown in Table 1. Compared to the non-NAFLD group, individuals of the NAFLD group were more possible to be older, male, diabetic, hypertensive, Mexican American, smoker, and had a lower education level. The NAFLD group also had higher levels of BMI, waist circumference, platelet, aminotransferase, alkaline phosphatase, gamma glutamyltransferase, fasting triglyceride, total cholesterol, high-density lipoprotein cholesterol, fasting glucose, hemoglobin A1c, and fasting insulin levels. However, marital status and poverty were not significantly different between the two groups.

### 3.2. Correlations between Urinary Phytoestrogen Concentrations and NAFLD

Table 2 shows the correlations between urinary phytoestrogen concentrations and NAFLD. In model 1 adjusted for other five phytoestrogens (tertiles), the urinary ENL concentration was negatively associated with NAFLD (OR of Tertile 2 : 0.72, 95% CI 0.57–0.92; OR of Tertile 3 : 0.46, 95% CI 0.33–0.65), while a positive correlation of urinary equol concentration with NAFLD was observed (OR of Tertile 2 : 1.30, 95% CI 1.01–1.65). When further considering demographic variables, we found that the results in model 2 (further adjusted for gender, age, race, education, marital status, and poverty) were concordant with the results in model 1. In model 3 (further adjusted for BMI, waist circumference, diabetes, smoking behavior, hypertension, total cholesterol, high-density lipoprotein cholesterol, fasting triglyceride), the correlation between the urinary equol concentration and NAFLD was no longer significant, while the concentration of urinary ENL was still inversely correlated with NAFLD (OR of Tertile 3 : 0.48, 95% CI 0.25–0.94).

### 3.3. Relations between Urinary Phytoestrogen Concentrations and NAFLD after Stratification by Gender or Age

Tables 3 and 4 further show the relations between urinary phytoestrogen concentrations and NAFLD stratified by gender and age, respectively. After adjusted for all confounding variables, a negative correlation of urinary ENL concentration and NAFLD was observed in males (OR of Tertile 2 : 0.39, 95% CI 0.17–0.86; OR of Tertile 3 : 0.43, 95% CI 0.19–0.95). Meanwhile, the urinary ENL concentration was inversely correlated to NAFLD in middle-aged adults (40–59 years) (OR of Tertile 3 : 0.29, 95% CI 0.10–0.83). While there were no significant associations between the urinary phytoestrogen concentrations and NAFLD in females, young adults (20–39 years), and older adults (60 years or over).

### 3.4. Relationships between NAFLD and the Urinary Phytoestrogen Concentrations after Stratification by Gender and Age

The relationships between NAFLD and the urinary phytoestrogen concentrations further stratified by different ages according to gender are shown in Table 5. In middle-aged males (40–59 years), the concentration of urinary equol was positively related with NAFLD in middle-aged males (OR of Tertile 3 : 4.27, 95% CI 1.02–17.85), while an inverse correlation was identified between the urinary ENL concentration and NAFLD (OR of Tertile 3 : 0.08, 95% CI 0.01–0.82). For elder males (60 years or over), the urinary concentration of END was inversely associated to NAFLD (OR of Tertile 2 : 0.18, 95% CI 0.05–0.69). However, there were no significant associations between the urinary phytoestrogen concentrations and NAFLD in other subgroups.

## 4. Discussion

To the best of our knowledge, this study based on NHANES data is the first to evaluate the association between urinary phytoestrogen concentrations and NAFLD. We found that urinary ENL concentration was negatively correlated to NAFLD. To be specific, a negative correlation between urinary ENL concentration and NAFLD was identified in males after stratification by gender, and in middle-aged adults, after stratification by age. When we further stratified the participants by different ages according to gender, the results showed that the ENL concentration was negatively correlated to NAFLD among middle-aged males, while the urinary equol concentration was positively correlated to NAFLD among middle-aged males. In addition, a negative correlation between END concentration and NAFLD was observed in elder males.

There is no epidemiological study on the relationship between lignans and NAFLD so far. However, some animal experiments have shown that lignans could reduce hepatic steatosis and regulate the related pathophysiological processes [29–31]. Studies by Fukumitsu et al. [29], Felmlee et al. [30], and Tominaga et al. [31] suggested that lignans reduced fatty acid synthesis by suppressing the expression of SREBP-1c, and finally decreasing hepatic fat accumulation [30, 31]. In addition, lignans also improved insulin resistance in mice by inducing the expression of adiponectin [29], which was also an important pathophysiological process of hepatic steatosis [57, 58]. A study in 2021 also showed that lignans could reduce liver steatosis score and NAFLD activity in rats [32]. These studies further support our finding that ENL was negatively correlated with NAFLD.

However, evidence of the relationship between lignans and NAFLD is still lacking, especially stratified by gender and age. Some studies have evaluated the relationship between lignans and obesity with metabolic disorders [59, 60], which are closely related to NAFLD. One study showed that elevated ENL levels were negatively correlated with obesity and components of the metabolic syndrome in males aged 20–60, but the relationship was not significant in elder males [61]. This is similar to our results observed in middle-aged males, but the difference was that we observed a negative correlation between middle concentration END and NAFLD in elder males. However, due to the lack of prior research studies, further comparisons were failed to be achieved.

A cross-sectional study which enrolled 115 postmenopausal women showed that women with high lignans intake had better metabolic status, including higher insulin sensitivity and lower obesity indexes [62]. However, the sample size of this study is too small and the selected population is relatively limited, so the conclusion needs to be confirmed in further researches. No significant relationships between lignans and NAFLD in females were observed in our study. The possible reason is that estrogen plays a critical role in inhibiting female hepatic lipid deposition [63–65], and lignans have both estrogen and antiestrogen effects in vivo [66], which means the role of lignans in female liver steatosis is unclear.

Some studies have shown that isoflavone additives and genistein can reduce liver steatosis and delay the progress of NAFLD [22–28]. A randomized controlled trial in 2018 revealed that insulin resistance and inflammatory status were improved after taking genistein supplementation in patients with NAFLD [28], but the included subjects were those already suffering from NAFLD, and instead of liver steatosis, insulin resistance and inflammatory status were selected as outcome variables. Additionally, in a 2013 trial, exercise training with isoflavone supplements could reduce the risk of NAFLD [67], but the subject included was only overweight postmenopausal women lacking a broad enough representation and the outcome was interfered by the confounding factor of exercise training. In our study, no significant correlation was observed between genistein, daidzein, O-DMA, and NAFLD. The difference in studies may be attributed to the different study populations and confounding factors included in the previous studies. In addition, the differences in demographic variables such as race, age, and personal economic conditions may also lead to differences from previous research studies. Our results showed that equol was positively correlated with NAFLD only in middle-aged males, but so far, there is no study on evaluating the relationship between equol and NAFLD directly. Equol is produced by microbe metabolism of ingested isoflavones in the intestine, but it varies greatly among different individuals [13, 17], which may also lead to the difference of the results. Therefore, further research is still needed to explore the relationship between isoflavones and NAFLD.

ENL and equol are estrogen analogs, but they have different affinities for different estrogen receptors (ER) [68, 69]; ENL has a high affinity for ER*α* [68], while equol has a high affinity for ER*β* [69]. Different ER has different effects on human health [70]. Specifically, ER*α* mainly mediates beneficial metabolic effects of estrogens such as improving glucose tolerance and insulin sensitivity, anti-lipogenesis, and reducing body weight [70]. By contrast, ER*β* plays an adverse role in insulin resistance and metabolic homeostasis of glucose and lipids [70]. Insulin resistance and metabolic disorders are the important mechanisms of NAFLD [71]. We speculate that the mechanism of the opposite effect of ENL and equol in NAFLD may be due to the activation of different ERs. However, there is still a lack of research on the direct relationship between equol and NAFLD, and further research studies and clinical tests are still required to confirm our hypothesis.

Our study has several strengths. First, our research was based on the NHANES database, which is designed by a complex stratified probability sampling and is generally representative in the American population. Second, our assessments of phytoestrogen were based on the concentrations of phytoestrogen in urine. The biomarkers of urine take into account the metabolic transformation of intestinal microbes, and therefore can reflect all food sources intake. As a result, the urinary phytoestrogen concentration can more accurately reflect the real and effective exposure. Third, this was the first epidemiological study on the relationship between single phytoestrogen and NAFLD. Only total isoflavones were focused on in previous studies, while individual differences of isoflavones have been ignored. Moreover, the relationship between lignans and NAFLD has not been studied up to now. Fourth, we considered the differences of age and gender for further stratified analysis. In addition, we adjusted demographic variables such as marital status, education level, and economic situation to control the potential confounding bias.

However, there are also some potential limitations in the current study. First, this is a cross-sectional study, which makes it impossible to infer the causal relationship between phytoestrogens and NAFLD. Second, the diagnosis of NAFLD was defined by USFLI, which was not verified histologically and was only calculated by a validated NAFLD prediction model. Therefore, the accuracy of NAFLD evaluation is relatively limited. However, on the other hand, liver biopsy in large observational studies is expensive and difficult to achieve. Third, urinary phytoestrogens in NHANES were determined using a single collection of urine. Although urinary phytoestrogen concentrations are reliable biomarkers of phytoestrogen intake [42–46], the single concentration possibly cannot accurately reflect long-term intake. However, fortunately, studies have shown that urinary phytoestrogens are relatively stable and significantly correlated with long-term dietary phytoestrogen intake [72–74]. Fourth, due to the limitation of sample size, it is difficult to further explore the ethnic differences in the relationship between phytoestrogen and NAFLD. Although the data of 6 cycles were included, the sample size of some subgroups was too small to lead to bias. Finally, further clinical controlled trials are still needed to explore the associations between phytoestrogens and NAFLD.

## 5. Conclusion

The present study suggests that in middle-age American males, the elevated urinary ENL concentration is negatively correlated to the risk of NAFLD, while the urinary equol concentration is positively correlated with NAFLD. Furthermore, a negative correlation between urinary END concentration and NAFLD was observed in elder American males. Therefore, individualized intake of phytoestrogens is preferred and may better treat and prevent NAFLD. More animal experiments are needed to explore the mechanism of the relationships between phytoestrogens and NAFLD, and further clinical randomized controlled trials are required to verify the current findings.

## Figures and Tables

**Figure 1:** Flowchart of the screening process of eligible participants from the National Health and Nutrition Examination Survey 1999–2010.

**Figure 2:** Calculation of the United States fatty liver index (USFLI).

**Table 1:** Weighted baseline characteristics of participants in the two groups.

Variables	Non-NAFLD (*n* = 1066)	NAFLD (*n* = 1228)	*P* value
Age (years)	40.2 ± 0.6	49.9 ± 0.6	<0.01
Sex (%)			
Male	38.6 (35.6–41.7)	59.5(56.3–62.6)	<0.01
Female	61.4 (58.3–64.4)	40.5 (37.4–43.7)	
Body mass index (kg/m^2^)	23.9 ± 0.1	33.7 ± 0.3	<0.01
Waist circumference (cm)	84.2 ± 0.4	111.9 ± 0.6	<0.01
Hypertension (%)	19.5 (16.9–22.5)	51.4 (47.7–55.0)	<0.01
Diabetes (%)	2.8 (1.9–4.1)	24.7 (21.8–27.8)	<0.01
Ethnicity (%)			
Non-Hispanic white	70.1 (66.5–73.5)	70.5 (65.9–74.7)	<0.01
Non-Hispanic black	15.5 (13.3–17.9)	6.5 (5.1–8.2)	
Mexican American	4.2 (3.2–5.5)	12.8 (10.3–15.7)	
Other Hispanics	3.8 (2.6–5.6)	6.0 (4.1–8.9)	
Others	6.4 (4.6–8.9)	4.2 (2.8–6.3)	
Smoking (%)			
Never	53.7 (49.7–57.7)	51.5 (47.0–56.0)	<0.01
Current smoker	26.1 (22.6–29.9)	18.0 (15.2–21.3)	
Ex-smoker	20.2 (17.2–23.6)	30.5 (27.0–34.3)	
High education (%)	64.3 (60.9–67.7)	51.1 (47.6–54.7)	<0.01
Marital status (%)	61.1 (57.6–64.6)	69.9 (66.3–73.2)	<0.01
Poverty (%)	11.1(9.0–13.5)	12.6 (10.4–15.2)	0.32
Platelet (10^9^/L)	257.5 ± 2.4	268.1 ± 2.3	<0.01
Albumin (g/dL)	4.3 ± 0.01	4.2 ± 0.01	<0.01
ALT (IU/L)	19.7 ± 0.3	32.6 ± 0.7	<0.01
AST (IU/L)	22.7 ± 0.3	27.0 ± 0.5	<0.01
ALP (IU/L)	61.9 ± 0.7	77.3 ± 1.1	<0.01
GGT (IU/L)	16.7 ± 0.4	44.2 ± 1.9	<0.01
Fasting triglyceride (mg/dL)	94.2 ± 2.3	195.2 ± 9.3	<0.01
Total cholesterol (mg/dL)	189.2 ± 1.6	203.8 ± 1.9	<0.01
HDL cholesterol (mg/dL)	59.8 ± 0.6	45.3 ± 0.4	<0.01
Fasting glucose (mg/dL)	92.8 ± 0.6	117.1 ± 1.4	<0.01
Hemoglobin A1c (%)	5.2 ± 0.02	5.9 ± 0.04	<0.01
Fasting insulin (pmol/L)	33.8 ± 0.5	130.9 ± 2.6	<0.01
Creatinine (mg/dL)	128.8 (122.4–135.2)	138.4 (132.6–144.2)	0.04
Daidzein (ng/mg Cr)	403.4 (290.2–516.5)	226.0 (174.3–277.7)	<0.01
O-DMA (ng/mg Cr)	135.8 (91.3–180.4)	55.2 (33.9–76.6)	<0.01
Equol (ng/mg Cr)	57.2 (26.1–88.4)	49.0 (13.9–84.1)	0.76
Enterodiol (ng/mg Cr)	141.0 (111.5–170.4)	172.6 (68.6–276.6)	0.56
Enterolactone (ng/mg Cr)	1049.8 (899.9–1199.8)	645.9 (506.8–785.1)	<0.01
Genistein (ng/mg Cr)	166.4 (121.2–211.5)	96.3 (76.1–116.6)	<0.01

Data are expressed as the weighted mean ± standard error or weighted frequency (95% confidence intervals). NAFLD: nonalcoholic fatty liver disease; ALT: alanine aminotransferase; AST: aspartate aminotransferase; ALP: alkaline phosphatase; GGT: gamma glutamyltransferase; HDL: high-density lipoprotein; O-DMA: O-desmethylangolensin; Cr: creatinine.

**Table 2:** Weighted ORs (95% CI) of NAFLD according to urinary phytoestrogen concentrations (tertiles).

Phytoestrogens (ng/mg Cr)	Model 1	Model 2	Model 3
Daidzein			
Tertile 1 (<24.92)	1.00	1.00	1.00
Tertile 2 (24.92 to <112.00)	0.95 (0.69–1.31)	1.00 (0.71–1.40)	0.76 (0.37–1.55)
Tertile 3 (≥112.00)	1.14 (0.72–1.80)	1.20 ( 0.74–1.96)	0.63 (0.22–1.77)
O-DMA			
Tertile 1 (<1.08)	1.00	1.00	1.00
Tertile 2 (1.08 to <10.59)	0.83 (0.64–1.08)	0.90 (0.66–1.21)	1.11 (0.61–2.02)
Tertile 3 (≥10.59)	0.73 (0.50–1.05)	0.79 (0.51–1.22)	1.21 (0.54–2.73)
Equol			
Tertile 1 (<4.00)	1.00	1.00	1.00
Tertile 2 (4.00 to <10.36)	1.30 (1.01–1.65)^*∗*^	1.36 (1.03–1.79)^*∗*^	1.64 (0.93–2.87)
Tertile 3 (≥10.36)	1.08 (0.81–1.44)	0.97 (0.69–1.37)	1.41 (0.71–2.80)
Enterodiol			
Tertile 1 (<23.96)	1.00	1.00	1.00
Tertile 2 (23.96 to <71.97)	1.03 (0.79–1.33)	0.98 (0.73–1.30)	0.89 (0.56–1.42)
Tertile 3 (≥71.97)	0.96 (0.73–1.24)	0.97 (0.71–1.31)	1.17 (0.65–2.09)
Enterolactone			
Tertile 1 (<187.38)	1.00	1.00	1.00
Tertile 2 (187.38 to <700.00)	0.72 (0.57–0.92)^*∗*^	0.57 (0.42–0.77)^*∗*^	0.63 (0.36–1.11)
Tertile 3 (≥700.00)	0.46 (0.33–0.65)^*∗*^	0.28 (0.19–0.41)^*∗*^	0.48 (0.25–0.94)^*∗*^
Genistein			
Tertile 1 (<12.00)	1.00	1.00	1.00
Tertile 2 (12.00 to <46.42)	0.93 (0.68–1.28)	0.86 (0.61–1.21)	1.19 (0.62–2.26)
Tertile 3 (≥46.42)	0.83 (0.59–1.18)	0.80 (0.56–1.15)	0.97 (0.41–2.24)

OR: odds ratio; CI: confidence interval; Cr: creatinine; O-DMA: O-desmethylangolensin. Model 1: adjusted for other five phytoestrogens. Model 2: additionally adjusted for gender, age, race, education, marriage, and poverty compared with model 1. Model 3: further adjusted for body mass index, waist circumference, smoking, diabetes, hypertension, triglycerides, total cholesterol, and high-density lipoprotein cholesterol on the basis of model 2. ^*∗*^*P* < 0.05.

**Table 3:** Weighted ORs (95% CI) of NAFLD according to urinary phytoestrogen concentrations (tertiles) stratified by gender.

Phytoestrogens (ng/mg Cr)	Model 1	Model 2	Model 3
Males			
Daidzein			
Tertile 1 (<24.92)	1.00	1.00	1.00
Tertile 2 (24.92 to <112.00)	0.98 (0.64–1.49)	0.91 (0.58–1.44)	0.54 (0.20–1.51)
Tertile 3 (≥112.00)	0.99 (0.51–1.92)	0.85 (0.40–1.80)	1.05 (0.25–4.44)
O-DMA			
Tertile 1 (<1.08)	1.00	1.00	1.00
Tertile 2 (1.08 to <10.59)	0.94 (0.64–1.36)	1.08 (0.72–1.64)	1.40 (0.55–3.55)
Tertile 3 (≥10.59)	0.87 (0.55–1.39)	1.05 (0.60–1.86)	0.93 (0.27–3.19)
Equol			
Tertile 1 (<4.00)	1.00	1.00	1.00
Tertile 2 (4.00 to <10.36)	1.55 (1.13–2.12)^*∗*^	1.72 (1.18–2.49)^*∗*^	2.17 (0.90–5.24)
Tertile 3 (≥10.36)	0.90 (0.60–1.37)	0.78 (0.48–1.28)	1.60 (0.55–4.63)
Enterodiol			
Tertile 1 (<23.96)	1.00	1.00	1.00
Tertile 2 (23.96 to <71.97)	1.24 (0.80–1.92)	0.98 (0.63–1.55)	1.12 (0.52–2.38)
Tertile 3 (≥71.97)	1.21 (0.81–1.82)	0.99 (0.64–1.53)	1.05 (0.52–2.12)
Enterolactone			
Tertile 1 (<187.38)	1.00	1.00	1.00
Tertile 2 (187.38 to <700.00)	0.63 (0.44–0.90)^*∗*^	0.44 (0.29–0.66)^*∗*^	0.39 (0.17–0.86)^*∗*^
Tertile 3 (≥700.00)	0.46 (0.30–0.71)^*∗*^	0.25 (0.15–0.41)^*∗*^	0.43 (0.19–0.95)^*∗*^
Genistein			
Tertile 1 (<12.00)	1.00	1.00	1.00
Tertile 2 (12.00 to <46.42)	0.84 (0.52–1.35)	0.81 (0.48–1.35)	1.47 (0.63–3.44)
Tertile 3 (≥46.42)	0.93 (0.53–1.66)	0.90 (0.48–1.68)	1.26 (0.42–3.82)
Females			
Daidzein			
Tertile 1 (<24.92)	1.00	1.00	1.00
Tertile 2 (24.92 to <112.00)	0.95 (0.60–1.50)	1.14 (0.68–1.89)	1.31 (0.43–4.00)
Tertile 3 (≥112.00)	1.36 (0.67–2.79)	1.75 (0.81–3.79)	0.62 (0.15–2.53)
O-DMA			
Tertile 1 (<1.08)	1.00	1.00	1.00
Tertile 2 (1.08 to <10.59)	0.75 (0.51–1.09)	0.75 (0.50–1.14)	0.77 (0.38–1.59)
Tertile 3 (≥10.59)	0.63 (0.36–1.11)	0.64 (0.34–1.19)	0.90 (0.35–2.32)
Equol			
Tertile 1 (<4.00)	1.00	1.00	1.00
Tertile 2 (4.00 to <10.36)	1.17 (0.82–1.66)	1.07 (0.72–1.59)	1.05 (0.54–2.01)
Tertile 3 (≥10.36)	1.34 (0.94–1.93)	1.13 (0.71–1.78)	1.20 (0.60–2.39)
Enterodiol			
Tertile 1 (<23.96)	1.00	1.00	1.00
Tertile 2 (23.96 to <71.97)	0.92 (0.63–1.33)	0.90 (0.58–1.41)	0.75 (0.35–1.59)
Tertile 3 (≥71.97)	0.89 (0.63–1.26)	0.88 (0.58–1.33)	0.99 (0.40–2.47)
Enterolactone			
Tertile 1 (<187.38)	1.00	1.00	1.00
Tertile 2 (187.38 to <700.00)	0.79 (0.54–1.15)	0.73 (0.48–1.10)	0.99 (0.46–2.12)
Tertile 3 (≥700.00)	0.46 (0.28–0.76)^*∗*^	0.31 (0.17–0.54)^*∗*^	0.54 (0.20–1.47)
Genistein			
Tertile 1 (<12.00)	1.00	1.00	1.00
Tertile 2 (12.00 to <46.42)	1.06 (0.70–1.59)	0.89 (0.57–1.39)	1.03 (0.40–2.68)
Tertile 3 (≥46.42)	0.83 (0.51–1.35)	0.69 (0.40–1.19)	0.75 (0.24–2.37)

OR: odds ratio; CI: confidence interval; Cr: creatinine; O-DMA: O-desmethylangolensin. Model 1 adjusted for other five phytoestrogens. Model 2 additionally adjusted for age, race, education, marriage, and poverty compared with model 1. Model 3 further adjusted for body mass index, waist circumference, smoking, diabetes, hypertension, triglycerides, total cholesterol, and high-density lipoprotein cholesterol on the basis of model 2. ^*∗*^*P* < 0.05.

**Table 4:** Weighted ORs (95% CI) of NAFLD according to urinary phytoestrogen concentrations (tertiles) stratified by age.

Phytoestrogens (ng/mg Cr)	Model 1	Model 2	Model 3
Age (20–39 years)			
Daidzein			
Tertile 1 (<24.92)	1.00	1.00	1.00
Tertile 2 (24.92 to <112.00)	1.09 (0.69–1.71)	1.23 (0.72–2.08)	1.32 (0.44–4.02)
Tertile 3 (≥112.00)	1.15 (0.61–2.15)	1.43 (0.68–3.04)	2.79 (0.50–15.67)
O-DMA			
Tertile 1 (<1.08)	1.00	1.00	1.00
Tertile 2 (1.08 to <10.59)	0.83 (0.50–1.38)	0.82 (0.49–1.37)	1.03 (0.35–3.08)
Tertile 3 (≥10.59)	0.89 (0.49–1.60)	0.97 (0.52–1.82)	1.90 (0.45–8.01)
Equol			
Tertile 1 (<4.00)	1.00	1.00	1.00
Tertile 2 (4.00 to <10.36)	1.39 (0.91–2.12)	1.68 (1.04–2.73)^*∗*^	1.19 (0.40–3.53)
Tertile 3 (≥10.36)	1.01 (0.62–1.62)	1.06 (0.60–1.88)	2.21 (0.56–8.77)
Enterodiol			
Tertile 1 (<23.96)	1.00	1.00	1.00
Tertile 2 (23.96 to <71.97)	0.94 (0.58–1.51)	0.87 (0.50–1.52)	1.11 (0.34–3.60)
Tertile 3 (≥71.97)	0.97 (0.58–1.65)	1.03 (0.56–1.92)	1.24 (0.26–5.86)
Enterolactone			
Tertile 1 (<187.38)	1.00	1.00	1.00
Tertile 2 (187.38 to <700.00)	0.62 (0.43–0.89)^*∗*^	0.48 (0.30–0.77)^*∗*^	0.39 (0.10–1.53)
Tertile 3 (≥700.00)	0.41 (0.24–0.71)^*∗*^	0.29 (0.16–0.55)^*∗*^	0.90 (0.25–3.25)
Genistein			
Tertile 1 (<12.00)	1.00	1.00	1.00
Tertile 2 (12.00 to <46.42)	0.88 (0.55–1.40)	0.89 (0.52–1.52)	0.47 (0.09–2.31)
Tertile 3 (≥46.42)	0.80 (0.48–1.34)	0.85 (0.46–1.58)	0.38 (0.06–2.29)
Age (40–59 years)			
Daidzein			
Tertile 1 (<24.92)	1.00	1.00	1.00
Tertile 2 (24.92 to <112.00)	0.88 (0.52–1.52)	0.83 (0.43–1.62)	0.62 (0.18–2.12)
Tertile 3 (≥112.00)	1.49 (0.65–3.43)	1.30 (0.54–3.10)	0.38 (0.09–1.55)
O-DMA			
Tertile 1 (<1.08)	1.00	1.00	1.00
Tertile 2 (1.08 to <10.59)	1.02 (0.61–1.69)	1.02 (0.58–1.81)	1.69 (0.51–5.54)
Tertile 3 (≥10.59)	0.56 (0.30–1.07)	0.56 (0.27–1.15)	1.16 (0.31–4.30)
Equol			
Tertile 1 (<4.00)	1.00	1.00	1.00
Tertile 2 (4.00 to <10.36)	1.02 (0.66–1.58)	1.10 (0.67–1.81)	2.35 (0.94–5.88)
Tertile 3 (≥10.36)	0.98 (0.61–1.57)	0.97 (0.55–1.70)	1.79 (0.60–5.32)
Enterodiol			
Tertile 1 (<23.96)	1.00	1.00	1.00
Tertile 2 (23.96 to <71.97)	1.10 (0.68–1.78)	1.16 (0.74–1.82)	0.72 (0.37–1.38)
Tertile 3 (≥71.97)	1.03 (0.63–1.68)	1.12 (0.66–1.89)	0.94 (0.38–2.33)
Enterolactone			
Tertile 1 (<187.38)	1.00	1.00	1.00
Tertile 2 (187.38 to <700.00)	0.65 (0.40–1.05)	0.63 (0.35–1.13)	0.50 (0.17–1.47)
Tertile 3 (≥700.00)	0.28 (0.16–0.50)^*∗*^	0.21 (0.12–0.39)^*∗*^	0.29 (0.10–0.83)^*∗*^
Genistein			
Tertile 1 (<12.00)	1.00	1.00	1.00
Tertile 2 (12.00 to <46.42)	0.92 (0.57–1.50)	0.79 (0.46–1.36)	1.35 (0.47–3.84)
Tertile 3 (≥46.42)	0.73 (0.38–1.37)	0.84 (0.45–1.57)	0.98 (0.35–2.74)
Age (≥60 years)			
Daidzein			
Tertile 1 (<24.92)	1.00	1.00	1.00
Tertile 2 (24.92 to <112.00)	0.83 (0.47–1.48)	0.85 (0.48–1.51)	0.77 (0.22–2.64)
Tertile 3 (≥112.00)	0.69 (0.28–1.71)	0.69 (0.28–1.74)	0.45 (0.08–2.52)
O-DMA			
Tertile 1 (<1.08)	1.00	1.00	1.00
Tertile 2 (1.08 to <10.59)	0.60 (0.35–1.02)	0.55 (0.32–0.96)	0.45 (0.16–1.31)
Tertile 3 (≥10.59)	0.80 (0.37–1.76)	0.88 (0.39–1.98)	0.84 (0.22–3.19)
Equol			
Tertile 1 (<4.00)	1.00	1.00	1.00
Tertile 2 (4.00 to <10.36)	1.65 (0.91–2.99)	1.32 (0.69–2.50)	1.74 (0.66–4.62)
Tertile 3 (≥10.36)	1.05 (0.59–1.89)	0.87 (0.46–1.64)	1.29 (0.55–3.05)
Enterodiol			
Tertile 1 (<23.96)	1.00	1.00	1.00
Tertile 2 (23.96 to <71.97)	0.71 (0.38–1.32)	0.70 (0.36–1.38)	0.57 (0.24–1.35)
Tertile 3 (≥71.97)	0.51 (0.29–0.88)^*∗*^	0.53 (0.29–0.97)	0.80 (0.32–2.01)
Enterolactone			
Tertile 1 (<187.38)	1.00	1.00	1.00
Tertile 2 (187.38 to <700.00)	0.81 (0.43–1.53)	0.73 (0.35–1.51)	0.92 (0.39–2.17)
Tertile 3 (≥700.00)	0.45 (0.25–0.84)^*∗*^	0.37 (0.19–0.72)^*∗*^	0.85 (0.29–2.52)
Genistein			
Tertile 1 (<12.00)	1.00	1.00	1.00
Tertile 2 (12.00 to <46.42)	1.20 (0.63–2.27)	1.08 (0.54–2.15)	1.35 (0.39–4.61)
Tertile 3 (≥46.42)	1.08 (0.46–2.54)	0.94 (0.39–2.28)	1.41 (0.32–6.33)

OR: odds ratio; CI: confidence interval; Cr: creatinine; O-DMA: O-desmethylangolensin. Model 1 adjusted for other five phytoestrogens. Model 2 additionally adjusted for gender, age, race, education, marriage, and poverty compared with model 1. Model 3 further adjusted for body mass index, waist circumference, smoking, diabetes, hypertension, triglycerides, total cholesterol, and high-density lipoprotein cholesterol on the basis of model 2. ^*∗*^*P* < 0.05.

**Table 5:** Weighted ORs (95% CI) of NAFLD across urinary phytoestrogen concentrations (tertiles) stratified by different ages according to gender.

Phytoestrogens (ng/mg Cr)	Males	Females
	Model 3	Model 3
Age (20–39 years)		
Daidzein		
Tertile 1 (<24.92)	1.00	1.00
Tertile 2 (24.92 to <112.00)	0.41 (0.02–9.89)	3.47 (0.48–25.26)
Tertile 3 (≥112.00)	2.71 (0.09–82.32)	1.17 (0.08–17.35)
O-DMA		
Tertile 1 (<1.08)	1.00	1.00
Tertile 2 (1.08 to <10.59)	2.18 (0.32–14.85)	0.37 (0.04–3.43)
Tertile 3 (≥10.59)	5.27 (0.32–86.63)	0.68 (0.06–7.80)
Equol		
Tertile 1 (<4.00)	1.00	1.00
Tertile 2 (4.00 to <10.36)	2.48 (0.35–17.46)	0.82 (0.07–9.09)
Tertile 3 (≥10.36)	1.40 (0.20–9.89)	3.89 (0.18–83.22)
Enterodiol		
Tertile 1 (<23.96)	1.00	1.00
Tertile 2 (23.96 to <71.97)	2.59 (0.19–35.56)	0.36 (0.07–1.82)
Tertile 3 (≥71.97)	0.15 (0.02–1.41)	0.83 (0.11–6.55)
Enterolactone		
Tertile 1 (<187.38)	1.00	1.00
Tertile 2 (187.38 to <700.00)	0.16 (0.01–2.42)	1.02 (0.23–4.61)
Tertile 3 (≥700.00)	0.93 (0.12–7.16)	6.71 (0.38–117.84)
Genistein		
Tertile 1 (<12.00)	1.00	1.00
Tertile 2 (12.00 to <46.42)	0.54 (0.10–2.78)	0.25 (0.01–4.69)
Tertile 3 (≥46.42)	0.88 (0.13–6.13)	0.11 (0.01–1.18)
Age (40–59 years)		
Daidzein		
Tertile 1 (<24.92)	1.00	1.00
Tertile 2 (24.92 to <112.00)	1.32 (0.21–8.24)	0.81 (0.19–3.45)
Tertile 3 (≥112.00)	0.63 (0.07–5.59)	0.45 (0.10–2.06)
O-DMA		
Tertile 1 (<1.08)	1.00	1.00
Tertile 2 (1.08 to <10.59)	6.12 (0.80–46.95)	1.10 (0.27–4.54)
Tertile 3 (≥10.59)	0.46 (0.08–2.77)	0.93 (0.26–3.29)
Equol		
Tertile 1 (<4.00)	1.00	1.00
Tertile 2 (4.00 to <10.36)	2.66 (0.66–10.70)	2.51 (0.65–9.65)
Tertile 3 (≥10.36)	4.27 (1.02–17.85)^*∗*^	0.91 (0.21–4.01)
Enterodiol		
Tertile 1 (<23.96)	1.00	1.00
Tertile 2 (23.96 to <71.97)	0.51 (0.14–1.88)	1.07 (0.38–3.02)
Tertile 3 (≥71.97)	0.59 (0.12–2.96)	0.80 (0.20–3.20)
Enterolactone		
Tertile 1 (<187.38)	1.00	1.00
Tertile 2 (187.38 to <700.00)	0.16 (0.02–1.52)	1.02 (0.22–4.67)
Tertile 3 (≥700.00)	0.08 (0.01–0.82)^*∗*^	0.39 (0.05–2.76)
Genistein		
Tertile 1 (<12.00)	1.00	1.00
Tertile 2 (12.00 to <46.42)	1.11 (0.22–5.60)	1.92 (0.47–7.83)
Tertile 3 (≥46.42)	1.82 (0.25–13.20)	0.76 (0.12–4.72)
Age (≥60 years)		
Daidzein		
Tertile 1 (<24.92)	1.00	1.00
Tertile 2 (24.92 to <112.00)	0.13 (0.01–1.28)	2.07 (0.28–15.51)
Tertile 3 (≥112.00)	0.32 (0.02–4.70)	0.62 (0.03–11.45)
O-DMA		
Tertile 1 (<1.08)	1.00	1.00
Tertile 2 (1.08 to <10.59)	0.47 (0.13–1.67)	0.29 (0.07–1.15)
Tertile 3 (≥10.59)	2.77 (0.45–16.94)	0.35 (0.05–2.50)
Equol		
Tertile 1 (<4.00)	1.00	1.00
Tertile 2 (4.00 to <10.36)	3.54 (0.76–16.39)	0.93 (0.26–3.30)
Tertile 3 (≥10.36)	0.96 (0.23–3.95)	1.16 (0.29–4.66)
Enterodiol		
Tertile 1 (<23.96)	1.00	1.00
Tertile 2 (23.96 to <71.97)	0.18 (0.05–0.69)^*∗*^	0.64 (0.13–3.23)
Tertile 3 (≥71.97)	1.10 (0.25–4.95)	0.73 (0.14–3.88)
Enterolactone		
Tertile 1 (<187.38)	1.00	1.00
Tertile 2 (187.38 to <700.00)	0.67 (0.17–2.59)	0.96 (0.25–3.63)
Tertile 3 (≥700.00)	0.94 (0.14–6.30)	0.86 (0.16–4.59)
Genistein		
Tertile 1 (<12.00)	1.00	1.00
Tertile 2 (12.00 to <46.42)	5.09 (0.45–57.91)	0.62 (0.07–5.44)
Tertile 3 (≥46.42)	2.18 (0.17–28.35)	0.86 (0.06–13.03)

OR: odds ratio; CI: confidence interval; Cr: creatinine; O-DMA: O-desmethylangolensin. Model 1 adjusted for other five phytoestrogens. Model 2 additionally adjusted for age, race, education, marriage, and poverty compared with model 1. Model 3 further adjusted for body mass index, waist circumference, smoking, diabetes, hypertension, triglycerides, total cholesterol, and high-density lipoprotein cholesterol on the basis of model 2. ^*∗*^*P* < 0.05.

## Data Availability

The data of this study were obtained from NHANES which are publicly available at https://wwwn.cdc.gov/nchs/nhanes/continuousnhanes/default.aspx.
